# Prevalence of coronary artery disease and its risk factors in Majmaah City, Kingdom of Saudi Arabia

**DOI:** 10.3389/fcvm.2022.943611

**Published:** 2022-09-08

**Authors:** Haitham M. Albar, Riyadh Ahmed Alahmdi, Abdulmalik A. Almedimigh, Riyaz Ahmed Shaik, Mohammad Shakil Ahmad, Abdulaziz Badar Almutairi, Waleed Khalid Z. Alghuyaythat, Shouq Yaseen Alaoufi, Worud Omar Aloyari, Rand Muslat S. Alanazi

**Affiliations:** ^1^Department of Surgery, College of Medicine, Majmaah University, Al Majmaah, Saudi Arabia; ^2^Department of Family Medicine, King Abdullah Bin Andulaziz University Hospital, Princess Nora Bint Abdulrahman University, Riyadh, Saudi Arabia; ^3^Department of Cardiac Surgery, Prince Sultan Cardiac Centre, Riyadh, Saudi Arabia; ^4^Department of Family and Community Medicine, College of Medicine, Majmaah University, Al Majmaah, Saudi Arabia; ^5^College of Medicine, Majmaah University, Al Majmaah, Saudi Arabia

**Keywords:** coronary artery disease, prevalence study, heart failure, risk factors, Saudi Arabia

## Abstract

**Objective:**

This study was carried out with an aim to outline the prevalence of coronary artery diseases, its risk of one region of the Saudi Arabia.

**Methods:**

A retrospective observational study conducted across five secondary medical centers located in the city of Majmaah. Hospital medical records and ministry of health records were screened over a 6-month period for data on patients admitted for Coronary artery disease (CAD). Data collected included sociodemographic characteristics, medical profile, and laboratory findings.

**Results:**

A total of 327 participants were included in this study with a median age of 64 and the majority being male participants (59.8%). The majority were married, held a primary school degree and earned a salary for living. A large number (82.9%) were hypertensive and diabetic (66.7%) and one-fourth had a previous MI (25.1%). A large number (73.7%) had heart failure with a mean ejection fraction of 44% (*SD* = 13). The causes of heart failure were mainly ischemic (56.3%) and hypertensive (28.1%). Readmission rates at 30 and 90 days then at 6 and 12 months were 22, 53.8, 68.8, and 75.8%, respectively. The mortality rates at the same time intervals were 5.5, 8.9, 14.1, and 22.9%, respectively. Predictors of readmission are age, CCI, and NYHA class.

**Conclusion:**

Coronary artery disease is the leading cause of heart failure. End stage CAD can have similar results in terms of readmission and mortality as heart failure. Future research should target patients in different stages of the condition and monitor their comorbidities which may impact the study findings.

## Background

Coronary artery disease (CAD) is a serious threat to societies as it is the leading cause of death in most countries of the world (1). With a 13% of death rates being due to CAD, the 2010 Global Burden of Disease Study identified it to be a modern pandemic (2). The death rate however is escalated to 21% in the MENA region with CAD being the number one cause of death (3). The prevalence of CAD is slightly higher among men than women in all age groups, however, there is a steep increase in prevalence as the age increases in both genders (4). The prevalence of CAD in the Kingdom of Saudi Arabia (KSA) was estimated to be 5.5% with slightly higher rates in urban areas when compared to rural areas (6 vs. 4.2%, respectively) (5, 6). The high cost of care has been a target in intervention studies (7) and these rates are similarly high in KSA to reach 40,164 Saudi Riyals per patient, equivalent to US $10,710 (8). The presented prevalence and cost number represent one region of the country with the lack of national studies that provide generalizability.

The risk factors associated with this condition can be general which apply to all nations, while others to be unique to one region of the world. Some of the unique risk factors of the Saudi region were identified to be dyslipidemia due to consumption of large amounts of Spanish coffee, sleep deprivation, and smoking especially among males (9). Despite that it was noted that the risk of developing coronary events in the coming 10 years was low in over 90% and high in 4% of the general population. However, the risk flared up to 26% in diabetic patients which makes diabetes to be a significant risk factor (10). On the other hand, the general risk factors were reported to be previous ischemic heart diseases, hypertension, smoking status, hyperlipidemia, DM, and family history of premature coronary artery diseases (10). Although at varying rates, these risk factors come in line with the international data (1). This local Saudi data was retrieved from the only national registry conducted in KSA as part of the Saudi Project for Assessment of Coronary Events (SPACE) in 2005 (11). No other updated registries have been conducted since then. Nationwide registries give insightful knowledge on the prevalence and the unique cultural risk factors of CAD in the country. This useful data can be used to inform policies and health care practices. The lack of such registries limits the capacities of policy making with data that is localized, sporadic, and lacking generalizability. Therefore, as a temporary replacement of national registries, a prevalence study on CAD was conducted in one large region of the Saudi Kingdom. An area of 30,000 square kilometers including five hospitals that care for a large population density. Therefore, the aim of this study was to outline the prevalence of coronary artery disease, its risk factors of one region of the Saudi Kingdom.

## Methods

### Observational study

This retrospective observational study was carried out in a secondary hospital in Majmaah Province, Saudi Arabia which is also a referral hospital for five primary and secondary medical centers located in the city of Majmaah. This city holds an area of 30,000 km^2^ with an area population density of 133,313 with more male than female inhabitants (77,822 vs. 55,491, respectively). The five hospitals are Hawtat Sudair, Prince Nasir Bin Saad Alsudairy hospital, Alartawijah Hospital, Tumair Hospital, and Al Zulfi Hospital.

### Procedure

Administrative and ethical approvals was granted from King Khalid Majmaah Hospital and from the Institutional Review Board, respectively. No patient consent was called for since no patient involvement was associated with the data collection. Additionally, data was deidentified and analyzed collectively. Administration approval was granted from each of the study hospitals and research teams were trained on data collection from the medical files of each facility. Hospital registries were scanned for patients presented with a confirmed diagnosis of coronary artery diseases in the last 6 months. Data on each of the eligible patients was then collected from the medical records of each hospital and mortality data was collected from the ministry records. Data collection took place between July and December 2021. Data is reflecting 7 years information retrospectively (from 2015 till 2022).

### Data retrieved included the below items

A. Sociodemographic characteristics including the age, gender, marital status, levels of education, occupation, family dependency, and smoking status.
B. Medical and surgical history including the comorbidities, implantable cardioverter defibrillator (ICD) or pacemaker inserted the Charlson comorbidity index (CCI) score and the ejection fraction for identifying those with heart failure among the sample in addition to the causes of heart failure when present.
C. Laboratory tests and vital signs upon admission and the New York Heart Association (NYHA) functional classification for those with heart failure. Length of hospital stay was also calculated from the admission and discharge dates of the patients.
D. Readmission and death data: this was retrieved from the Ministry of Health records and compared to the time of discharges, which was retrieved from the hospital medical records.

### Data analysis

Data was entered into Microsoft Excel^®^ 2007 and the EPI INFO 7 for data analysis. Univariate data was presented as frequencies and percentages when categorical and as medians and interquartile ranges or as means and standard deviation (*SD*) when continuous. Multivariate analysis was done to predict readmission of patients at 30 days using variables that were mostly significant in the international literature.

## Results

A total of 327 patients' data were collected in the 6-month study period. The median age of the study participants was 64 years (interquartile range 56–74) with the majority (59.6%) being male participants. The majority (78.9%) were married and less than half (40.4%) gained no more than primary school education with 12.2% being illiterate. A large number (85%) had a paid job and more than 40% had a spouse depending on them financially and 47.7 had a child in their dependency. More than half (55.7%) smoked and only 1.8% of the sample consumed alcohol. The sociodemographic characteristics are presented in Table 1.

**Table 1:** Baseline and demographic characteristics of the study participants (*N* = 327).

**Variables**	**Frequency (%)**
**Demographic characteristics**
Age^**a**^	64 (56–74)
Female	132 (40.4)
**Marital status**
Single	51 (15.6)
Married	258 (78.9)
Divorced/Widowed	18 (5.5)
**Level of education**
No education	40 (12.2)
Primary	132 (40.4)
Secondary	97 (29.7)
University	58 (17.7)
**Occupation**
Salaried	278 (85.0)
Retired/Unemployed	49 (15.0)
**Family dependency**	
Wife/Husband	137 (41.9)
Daughter/Son	156 (47.7)
Other	34 (10.4)
**Habits**
Smoke	182 (55.7)
Drink	6 (1.8)

^*a*^Variables expressed in median and interquartile range.

In terms of comorbidity, a large number (82.9%) were hypertensive, more than two-thirds (66.7%) were diabetic, only 25.1% had a previous history of MI and 44.6% were either asthmatic or had chronic obstructive pulmonary disease. A large number of the participants (73.7%) had heart failure with a mean ejection fraction of 44% (*SD* = 13). The causes of heart failure were documented to be ischemic in 56.3% and hypertensive in 28.1% of the cases. Data of the comorbidities are presented in Table 2.

**Table 2:** Comorbidity conditions and causes of heart failure.

**Variables**	**Frequency (%)**
**Comorbidities**
HTN	271 (82.9)
DM	218 (66.7)
MI	82 (25.1)
Peripheral vascular disease	46 (14.1)
COPD/Asthma	146 (44.6)
ICD/Pacemaker	33 (10.1)
Chronic HF cases	241 (73.7)
CCI score^a^	4.86 (2.21)
EF^a^	44 (13)
**Cause of HF**
Ischemia	184 (56.3)
HTN	92 (28.1)

^*a*^Variables expressed in mean and standard deviation.

The mean hemoglobin level was 11.74 (*SD* = 3.21), mean creatinine was 1.85 (*SD* = 0.59), and mean albumin was 3.38 (*SD* = 0.38). The median cholesterol level was 162 (quartile range = 124–176) and median pro-BNP was 1,953. The mean heart rate upon presentation was 86 (*SD* = 18), mean systolic blood pressure (SBP) was 142 (*SD* = 24), and the mean diastolic blood pressure was 80 (*SD* = 15). The median length of stay was 15 days. Details of the laboratory findings and the vital signs are presented in Table 3.

**Table 3:** Laboratory investigations, physiological, and other parameters.

**Variables**	**Frequency (%)**
**Laboratory investigations**
Hgb^a^	11.74 (3.21)
Creatinine^a^	1.85 (0.59)
Albumin^a^	3.38 (0.38)
Cholesterol^b^	162 (124–176)
Pro-BNP^b^	1,953 (1,756–2,234)
Gamma GT^b^	44 (34–58)
**Vital signs**
HR^a^	86 (18)
SBP^a^	142 (24)
DBP^a^	80 (15)
**Length of stay** ^**b**^	**15 (6–25)**

^*a*^Variables expressed in mean and standard deviation.

^*b*^Variables expressed in median and interquartile range.

Considering the large number of patients with heart failure, The NYHA functionality classification was shown to be 14.1, 25.7, 32.4, and 27.8% for classes I, II, III, and IV, respectively, as presented in Table 4.

**Table 4:** New York Heart Association functional classification (NYHA).

**Variables**	**Frequency (%)**
***NYHA***
Class-I	46 (14.1)
Class-II	84 (25.7)
Class-III	106 (32.4)
Class-IV	91 (27.8)

In terms of readmission, it was noted that 22% of the sample were readmitted within 30 days, 53.8% were readmitted within 90 days, 68.8% were readmitted within 6 months, and 75.8% were readmitted within the year. The death rates however at these time intervals were 5.5, 8.9, 14.1, and 22.9% respectively. These details are presented in Table 5.

**Table 5:** Readmissions and death.

**Variables**	**Frequency (%)**
**Readmission**
30 days	72 (22.0)
90 days	176 (53.8)
6 months	225 (68.8)
12 months	248 (75.8)
**Death**
30 days	18 (5.5)
90 days	29 (8.9)
6 months	46 (14.1)
12 months	75 (22.9)

Logistic regression analysis was conducted to produce a model for predicting readmission in patients with CAD. Since a large number of the patients had heart failure and considering this condition will be associated with frequent readmission, the NYHA class was added to the model along with age and the CCI. The model showed these variables to be significantly associated with readmission where increasing age and higher scores on the CCI doubled and tripled the risk of readmission when compared to younger ages and lower CCI scores. Additionally, it was noted that those with NYHA class III and IV were two times more likely to be readmitted than their counterparts with lower NYHA classes. The details of this analysis are presented in Table 6.

**Table 6:** Logistic regression analysis for predicting risk factors associated with readmission of patients at 30 days.

**Factors**		**Odds ratio**	**95% Confidence interval**	***P*-value**
Age		2.14	(1.44–5.76)	0.044
CCI		3.76	(2.88–6.17)	0.006
NYHA	Class I (Ref)	1	–	–
	Class II	1.80	(1.06–2.69)	<0.001
	Class III	2.39	(1.13–5.07)	<0.001
	Class IV	2.06	(1.40–3.53)	<0.001

## Discussion

This study aimed to outline the prevalence of coronary artery diseases, its risk factors of one region of the Saudi Kingdom. The results showed that the cohort had a long history of CAD leading to heart failure which impacted the readmission rates. The rates are in turn comparable to heart failure readmissions in the international literature and higher than readmissions related to CAD (12). Additionally, heart failure readmission and mortality rates at 12 months were significantly higher among CAD patients when compared to non-CAD patients (13). Albeit, heart failure readmission rates at 30 days have been reported to go as high as 39% in the same study country (14).

On the other hand, CAD is also highly prevalent among patients with heart failure as it is the primary cause of the latter condition in more than two-third of the cases (15). Additionally, up to 66% of those with preserved ejection fraction heart failure have some form of vascular coronary ischemia (16). Among CAD patients, those who had reduced ejection fraction had higher in-hospital mortality (13). In the current study, more than 70% of the study participants had HF and more than half had a functional class of III or IV which shows that the readmission rates are not completely specific to CAD. This was also seen in a study on 15 Swiss and German centers where readmission and death rates combined were high at 30 (11%) and 90 days (26%), and the reason was HF in 33% of the incidents, all other cardiovascular problems in 32%, and non-cardiovascular problems in 45% (17). Also, knowing that CAD is the leading cause of heart failure, a study showed high overall prevalence of CAD among HF patients with a reported prevalence of 60.2% in seven Middle Eastern countries, and 62.5% in Saudi Arabia specifically (13). A study conducted in Lebanon showed that 73.61% of readmissions were due to heart failure exacerbation with CAD being a significant predictor of readmission (18). Moreover, the numbers of patients with NYHA class III and IV among the CAD group was relatively high in comparison to a previous international study assessing the characteristics of patients with CAD in several countries of the world. This study showed the class III and IV among the CAD patients to be 13% and 2% globally (1). These changes may be accounted for by the large number of patients with heart failure in this group or in KSA in general.

Coronary artery disease is the leading single reason of mortality and loss of Disability Adjusted Life Years (DALYs) internationally, 7 million deaths and 129 million DALYs yearly where most of which come from low- and middle-income countries, especially in Latin America and the Middle East (3). The death rates in our study were 5.5% within 30 days and 22.9% within a year which fell within the ranges provided through an international review. This review showed mortality rates for patients with both CAD and HF to range between 4.9% and 12.3% at 30 days with lower rates to reach 1.3% with coronary interventions. This same study reported the mortality rates at 1 year to range between 13.7% and 38% (19). On the other hand, when looking at HF mortality alone, a study in Saudi Arabia showed these rates to be 15.8% within 30 days and 12.1% within 90 days (14).

To compare between HF patients with CAD or without CAD in some Middle Eastern countries, Salam et al. conducted a study and found that there were no significant differences at 3 months between the two groups in regard to mortality rates (13). However, the mortality rates at 12 months were significantly greater among CAD when compared to non-CAD patients. Also, at 1 year the mortality rates were significantly variable.

The limitations of the study lie first in the design which restricts the study to the available data. The main limitation of the current study, however, is the high rates of patients with heart failure which prevented the isolation of the readmissions to the CAD causes. This is even more dramatic with the high numbers of patients having poor functional classes (Class II and IV). Therefore, future studies should exclude those with heart failure to isolate the causes of readmissions to CAD only. Alternatively, registries can be of long duration to capture all patients with CAD with and without HF with larger sample size and a broader setting within the region and country. This will allow the analysis of these rates at the different stages of the condition and to find the actual prevalence of the disease. Moreover, in the future using of artificial intelligence across all population may give an insight to the predicted prevalence and associated risk factors and that will be of great use as well.

In this level of study we can increase the level of awareness for the physician in PHC in those five hospital about how to manage such cases like post CAD who have CHF or HTN through directed workshops or seminars.

## Conclusion

This study outlined the prevalence and risk factors of CAD in one large region of the Saudi Kingdom. The results revealed higher rates than those found in the international literature for having a large number of patients with heart failure within the sample. Although CAD is the leading cause of heart failure, end stage CAD can have similar results in terms of readmission and mortality as heart failure. Future research should target patients in different stages of the condition and monitor their comorbidities which may impact the study findings.

## Data availability statement

The original contributions presented in the study are included in the article/Supplementary material, further inquiries can be directed to the corresponding author/s.

## Author contributions

Conceptualization: HA, RAA, and AAA. Methodology: RS and MA. Software: SA. Formal analysis: RS. Resources: MA, HA, and RMA. Data collection: ABA, WKA, SA, WOA, and RMA. Writing-original draft preparation: HA, RAA, and RS. Supervision, project administration, and validation: HA. All authors contributed to the article and approved the submitted version.

## Funding

The authors would like to thank the Deanship of Scientific Research at Majmaah University for funding this study with project number R-2022-259.

## Conflict of interest

The authors declare that the research was conducted in the absence of any commercial or financial relationships that could be construed as a potential conflict of interest.

## Publisher's note

All claims expressed in this article are solely those of the authors and do not necessarily represent those of their affiliated organizations, or those of the publisher, the editors and the reviewers. Any product that may be evaluated in this article, or claim that may be made by its manufacturer, is not guaranteed or endorsed by the publisher.
